# Analysis of the Effect of Posterior Lateral Malleolus Plate Fixation on the Curative Effect and Mechanical Stability of Complex Ankle Fractures

This article has been retracted.

**DOI:** 10.1155/2022/7101007

**Published:** 2022-06-06

**Authors:** Junpu Zha, Guolei Zhang, Jingtao Zhang, Xiaoqing Wang, Jie Li, Jun Di

**Affiliations:** ^1^Department of Orthopedics, The Third Hospital of Hebei Medical University, Shijiazhunag 050052, China; ^2^Department of Obstetrics, Hebei General Hospital, Shijiazhuna 050055, China

## Abstract

This paper investigates the effect of lateral and posterior 1/3 tubular plate bone plate fixation on the curative effect, wound healing, and mechanical stability of complex ankle fracture. 80 patients with complex ankle fractures treated in our hospital from January 2018 to July 2020 are selected for the study, and 80 patients are randomly divided into posterior fixation group and lateral fixation group according to the number table method, with 40 patients in each group. Patients in the posterior malleolus fixation group are treated with posterior lateral malleolus plate fixation, and patients in the lateral malleolus fixation group are treated with lateral malleolus plate fixation. The differences in efficacy, mechanical stability, wound healing, visual analog scale (VAS) pain score, and American Association of Foot and Ankle Surgery (AOFAS) ankle function are compared. The subjects are followed up for 6 months until January 2022. In patients with complex ankle fracture, 1/3 tubular plate osteoplate fixation in the posterior lateral malleolus can improve clinical efficacy and mechanical stability, which is helpful to promote incision healing and reduce the risk of complications. The 1/3 tubular plate osteoplate fixation in the posterior lateral malleolus is worthy of clinical promotion and application.

## 1. Introduction

In recent years, with the continuous improvement of transportation tools and living standards, the incidence of traffic accidents and the risk of joint fracture are increasing year by year. Among them, ankle fracture is a relatively common intra-articular fracture, which poses a certain threat to patients' quality of life and health [1]. The ankle joint is the joint with the largest weight bearing in the human body. The structure of the joint is special and diverse, and the complex ankle fracture is characterized by obvious complexity. The adoption of strong internal fixation is of great significance to improve the clinical efficacy of ankle fracture and prevent complications [2]. Although traditional fixation materials such as steel wire and Kirschner wire can achieve certain fixation effect, they have disadvantages such as poor stability and poor antirotation ability. Therefore, it is an urgent problem to explore a new fixation scheme for lateral malleolus fracture [3]. 1/3 tubular plate is a common clinical material for fracture fixation in recent years. It has the advantages of high stability and strong antirotation ability and has achieved certain results in clinical orthopedic fixation. However, traditional lateral fixation of lateral malleolus fibula will cause incision infection and malunion and other complications, which is not conducive to postoperative recovery of patients. The posterior fibula is a new choice for 1/3 tubular plate fixation, which can reduce the risk of wound infection and promote wound healing [4]. Therefore, the posterolateral and posterolateral lateral malleolus tubes are applied, respectively. The effects of plate osteoplate fixation on clinical efficacy, incision healing, and mechanical stability of patients with complex ankle fracture provide reference for clinical treatment plan optimization and treatment safety of patients with complex ankle fracture.

A total of 80 patients with complex ankle fractures treated in our hospital from January 2018 to July 2020 are selected for the study. According to the number table method, 80 patients are randomly included in the posterior fixation group and lateral fixation group, with 40 patients in each group. There are 40 cases in the study group, including 30 males and 10 females, aged from 20 to 58 years old with an average of (44.32 ± 10.98) years old. There are 20 cases of traffic injury, 14 cases of fall injury, and 6 cases of falling injury. A total of 40 patients are included in the conventional group, including 28 males and 12 females, aged from 21 to 59 years, with an average of (43.28 ± 11.10) years, including 22 traffic injuries, 12 falls, and 6 falls. There is no significant difference in the baseline data between the two groups and a valid comparison could be made (*P* > 0.05). This research procedure has been approved by our school (ethics batch number: TJ-IRB20171212).

Inclusion criteria include as follows: (1) unilateral fracture; (2) it is consistent with the diagnostic criteria of complex ankle fracture and confirmed by CT imaging [5]; (3) the time to hospital treatment for fracture ≤10 days; (4) no contraindications or obvious allergic reactions; (5) no malignant pathologic fracture such as primary or metastatic tumor; (6) patients and their families voluntarily signed informed consent and confidential documents after knowing the study contents in detail. Exclusion criteria include as follows: (1) there is a history of active infection or thrombosis or cerebral infarction; (2) suffering from inflammatory joint diseases such as arthritis and rheumatoid arthritis of the hip; (3) with a history of cognitive impairment such as Parkinson's disease or hemiplegia or other mental diseases; (4) participate in other research and experiment in the same period.

The remainder of this paper is organized as follows.  Section 2 describes related work.  Section 3 presents the experimental method.  Section 4 provides the experimental result. Finally, the discussion and conclusion of this study are given in Section 5.

## 2. Related Work

Ankle joint is the joint with the largest weight bearing in the human body, and the posterior ankle has an important influence on the stability of the ankle joint and physiological functions such as human walking [6]. The integrity of the ankle point structure is the key to maintaining the stability of the ankle joint. However, the reduction, fixation, and fibula recovery of lateral malleolus fracture treated by manual reduction or open reduction, and internal fixation cannot achieve the expected effect and has no significant effect on the anatomic reduction and stability of the ankle joint [7]. The traditional application of single screw fixation can play the role of compression at the broken end, but the weakness of this method lies in its low stability and antirotation ability. Although tension band steel wire has antirotation ability, it has a high risk of wire fracture, which may cause serious complications, leading to poor safety [8]. Tubular steel plate is a new fixation material with good fixation and antirotation ability and is not easy to break. Its application effect in ankle joint fixation has been certified, but the fixation plate at different positions of lateral malleolus has a certain influence on the clinical efficacy and joint stability of joint fixation [9]. Some studies believed that although the lateral fibular fixation plate could achieve a certain fixation effect, the risk of poor postoperative incision healing is relatively high, and the safety of this plan is relatively poor [10]. In addition, it can reduce the risk of wound infection and further promote wound healing and physical recovery of patients. Thus, the stability of joint fixation is reduced, and the risks of plate fracture, fracture dislocation, and healing malformation are increased. In addition, the 1/3 tubular plate used for fixation at the lateral part of the lateral malleolus, which covers relatively little soft tissue, is prone to incision cracking and complications of plate exposure, thus increasing the risk of incision infection. In external ankle back application type, the tube plate fixed has some advantages. For example, it effectively reduces the risk of failure and postoperative fixed plate fracture. Ultimately, it plays a positive role in promoting wound healing and improving clinical efficacy.

Far from the direct impact of articular surface displacement on ankle fixation and recovery, large displacement leads to the reduction of ankle tolerance. Although the application of preoperative stress test is less, the results obtained by simulating fibula stress displacement test have high accuracy in the evaluation of ankle fracture stability. Therefore, the stress test is used to evaluate stability as a good indicator of ankle joint efficacy, which has a certain reference value. It suggests a third pipe steel slabs external ankle back for bone plate fixation can obtain a higher fixation effect. It can enhance joint stability and function after fixation and reduce joint pain. Analysis of the reason may be composed of ligament of soft tissue. The bone stable ankle structure is mainly composed of middle stable structure, which provides stability. The bone stable ankle joint structure mainly includes the attachment points between the fibular joint ligaments, ligaments and bone slices, behind the ankle joint ligaments and behind the fibular tibiofibular transverse ligaments. The risk of talus displacement will be reduced after the stability of the ankle joint recovers well. Therefore, the effective reduction and fixation of the ankle joint through a 1/3 tubular steel plate can reduce the compression and injury of the talus joint caused by ankle fracture displacement. It helps to reduce the weight bearing of the ankle joint, improve the stability of the posterior joint, and effectively reduce and enhance the ankle function of patients.

## 3. The Proposed Method

Patients in the posterior fixation group are treated with posterior lateral malleolus plate fixation, and the specific procedures are as follows: in the supine position, combined subepidermal anesthesia is performed, the affected limb is treated with an inflated tourniquet, and the specific location of the fracture is determined by CT examination before surgery. With the fibula fracture line as the midpoint, a posterior approach arc incision is made at 9.0 cm outside the sural nerve, and the skin and subcutaneous tissues are separated one by one so that the fibula fracture ends are completely exposed. After the reduction of lateral malleolus fracture, the tubular plate is placed on the lateral fibula for fixation. The deep fascia is cut, and the peroneus longus support band is cut to completely expose the peroneus longus tendon and flexor hallux longus tendon and pull them laterally and medially, respectively. After the posterior fracture is completely exposed, the fracture block is reduced under direct vision. The c-arm X-ray machine is used to confirm the reduction, and a supporting 1/3 tubular plate is inserted for fixation. After the internal fixation position is determined again, the negative pressure drainage tube is indignant, and the incision is sutured layer by layer. After surgery, antibiotics are given and ankle exercises are performed 24 hours after surgery to avoid weight-bearing activities of the affected limb within 6 weeks after surgery. Patients in the lateral fixation group are treated with lateral malleolus plate fixation, which is fixed on the lateral side of the fibula, and other operations are the same as those in the posterior fixation group. Patients in both groups are followed up for 6 months, and the end date of follow-up is January 2022. The time points of follow-up are 1 month, 3 months, and 6 months after surgery, and the preoperative time points and the above time points are denoted as T1–T4.

The clinical efficacy of the patients is calculated and the difference is compared. The criteria are as follows: (1) the joint function score is above 90, the pain sensation disappeared completely, and the patients could walk normally. The joint function score ranged from 75 to 89, the pain is significantly reduced, and the patients could walk without the help of others. The joint function score is within 50∼74, the pain is relieved, and walking with the assistance of others is effective. If the joint function score is lower than 50, the pain is not significantly alleviated or aggravated, and the inability to walk without help is considered invalid. The total effective rate = (cured + effective + effective)/total number of cases × 100% [11]. (2) Incision healing time and hospitalization time of 80 subjects are recorded and divided into groups. (3) External rotation stress test is used to evaluate and compare the postoperative ankle joint stability. After the external fixation of the external ankle fracture is wrapped with stress on the C-arm X-ray machine, the fluoroscopy test is carried out. After one hand fixes the tibia, the other hand twists the eversion stress outward on the foot, holds the caliper leg respectively at the fracture site outside the ankle, reads the applied stress and the applied stress meter, and the deviation. In order to avoid the data value, the assistant reads it. The size of the fibular displacement is determined according to the difference between the readings. If the size of the fibular displacement is more than 1 mm, it is considered as positive in the external rotation stress test; otherwise, it is negative [12]. (4) visual analogue scale (VAS) is used to evaluate the pain degree of patients before surgery, 1 month, 3 months, and 6 months after surgery for comparison. A piece of white paper with a scale of 0∼10 is taken and arbitrarily marked on the paper by patients according to their own pain. The total score is 0∼10 points. The pain degree of patients increased with the increase of the score [13]. (5) use the American Orthopaedic Foot and Ankle Society (AOFAS) ankle exercises. The ankle function of patients at different time points is evaluated by the energy scale, and the differences are compared. The scale included five dimensions of muscle strength, range of motion, walking function, pain, and ankle stability and mobility. The total score is 100 points, and the ankle function increased with the increase of the score [14]. (6) The difference in the incidence rate of wound infection, malunion, and plate fracture in each group is recorded and compared.

The SPSS 24.0 software is used to process the data in the study. The counting data are represented by the *χ*^2^ test, the measurement data are represented by *t*-test, the mean ± standard deviation ($\bar{x}\pm s$), and the multiple groups of the data are represented by the *F* test. Mauchly test is used to compare the data at different time points within the group. *P* > 0.05 indicated that the covariance matrix is full of football symmetry, and *P* < 0.05 indicated that the difference is statistically significant.

## 4. The Experimental Results

### 4.1. Comparison of Curative Effect Gap after Fixation

The total clinical response rate of the posterior fixation group is higher than that of the lateral fixation group, and the data difference is statistically significant (*P* < 0.05).  Table 1 is the total clinical response rate gap.

### 4.2. Comparison of Perioperative Clinical Indicators

Compared with the lateral fixation group, the length of hospital stay, and incision healing time of the posterior fixation group are significantly shortened, and the data differences are statistically significant (*P* < 0.05).  Table 2 shows the differences in perioperative clinical indicators.

### 4.3. Comparison of Ankle Function Gap at Different Time Points

AOFAS scores show an increasing trend in both groups, and the scores of posterior fixation group are higher than those of the lateral fixation group at three postoperative time points, with statistically significant differences (*P* < 0.05).  Table 3 presents the ankle function differences at different time points.  Figure 1 provides the difference in ankle function at different time points.

### 4.4. Difference in Stability Results of External Rotation Stress Test after Operation

The positive rate of external rotational stress stability in the posterior fixation group is lower than that in the lateral fixation group (17.50% and 37.50%, respectively), and the difference is statistically significant (*χ*^2^ = 4.013, *P*=0.045).  Figure 2 is the CT images of the posterior fixation group before and after surgery.

### 4.5. Difference in Pain Degree at Different Time Points

VAS scores in both groups show a decreasing trend, and scores in the posterior fixation group are significantly lower at three postoperative observation time points, with statistically significant differences (*P* < 0.05).  Table 4 presents the difference in pain degree at different time points.  Figure 3 is the difference in pain degree at different time points.

There are 4 cases of incision infection in the posterior fixation group, 8 cases of incision infection and 5 cases of plate fracture in the lateral fixation group. The incidence of complications in the lateral fixation group is higher, 10.00% and 32.50%, respectively, with statistically significant differences (*χ*^2^ = 6.050, *P*=0.014).

## 5. Discussion and Conclusion

There are still some limitations in this study. For example, fewer than 100 cases are included in the paper during a long study period, resulting in a relatively small number of study samples, which may lead to research data bias. Therefore, more eligible study samples should be screened in multiple medical centers for large-sample, multicenter in-depth studies.

In conclusion, posterior lateral malleolus tubular plate osteoplate fixation can improve the clinical efficacy and mechanical stability of patients with complex ankle fractures. At the same time, this method can promote the wound healing of patients, which is a good fixation plan that can be popularized and applied in clinic.

## Figures and Tables

**Figure 1:** Difference in ankle function at different time points.

**Figure 2:** CT images of the posterior fixation group before and after surgery.

**Figure 3:** Difference in pain degree at different time points.

**Table 1:** Total clinical response rate gap (*n*(%)).

Group	Cure	Excellence	Effective	Invalid	Total effective rate
Rear fixed group (*n* = 40)	8 (20.00)	14 (35.00)	14 (35.00)	4 (10.00)	36 (90.00)
External fixed group (*n* = 40)	6 (15.00)	10 (25.00)	12 (30.00)	12 (30.00)	28 (70.00)
*x* ^2^					5.000
*P*					0.025

**Table 2:** Differences in perioperative clinical indicators ($\bar{x}\pm s$).

Group	HOD (d)	Incision healing time (d)
Rear fixed group (*n* = 40)	8.54 ± 2.43	8.38 ± 2.23
External fixed group (*n* = 40)	17.62 ± 2.74	16.71 ± 2.67
*t*	−15.681	−15.144
*P* value	<0.001	<0.001

**Table 3:** Ankle function differences at different time points (*x* ± *s*).

Group	Time point	AOFAS grade
Rear fixed group (*n* = 40)	T1	43.54 ± 2.53
	T2	66.52 ± 3.34
	T3	79.26 ± 4.66
	T4	92.03 ± 5.44
External fixation group (*n* = 40)		
	T1	43.49 ± 2.28
	T2	55.52 ± 2.34
	T3	67.26 ± 3.46
	T4	85.03 ± 4.84
*F*_timepoint_		416.542
*P*_timepoint_		<0.001
*F*_point∗group_		534.334
*P*_point∗group_		<0.001

**Table 4:** Difference in pain degree at different time points (*x* ± *s*).

Group	Time point	VAS grade
Rear fixed group (*n* = 40)	T1	6.54 ± 2.33
	T2	4.52 ± 2.14
	T3	3.24 ± 1.87
	T4	2.03 ± 1.24
External fixation group (*n* = 40)		
	T1	6.56 ± 2.31
	T2	5.62 ± 2.21
	T3	4.31 ± 1.90
	T4	3.33 ± 1.53
*F*_timepoint_		452.312
*P*_timepoint_		<0.001
*F*_point∗group_		434.315
*P*_point∗group_		<0.001

## Data Availability

The simulation experiment data used to support the findings of this study are available from the corresponding author upon request.
